RETRACTED

# Investigating the Possibility of Green Synthesis of Silver Nanoparticles Using *Vaccinium arctostaphlyos* Extract and Evaluating Its Antibacterial Properties

**DOI:** 10.1155/2021/5572252

**Published:** 2021-05-03

**Authors:** Sedighe Khodadadi, Nafiseh Mahdinezhad, Bahman Fazeli-Nasab, Mohammad Javad Heidari, Baratali Fakheri, Abdolhossein Miri

**Affiliations:** ^1^Department of Biotechnology and Plant Breeding, Faculty of Agriculture, University of Zabol, Zabol, Iran; ^2^Research Department of Agronomy and Plant Breeding, Agricultural Research Institute, University of Zabol, Zabol, Iran; ^3^Department of Biotechnology and Plant Breeding, Faculty of Agriculture, Ferdowsi University of Mashhad, Mashhad, Iran; ^4^Faculty of Pharmacy, Cyprus International University, Lefkosa, Turkish Republic of Northern Cyprus, Lefkosa, Cyprus; ^5^Department of Pharmacognosy, School of Pharmacy, Zabol University of Medical Sciences, Zabol, Iran

## Abstract

**Objective:**

Vaccinium genus plants have medicinal value, of which *Vaccinium arctostaphylos* (Caucasian whortleberry or Qare-Qat in the local language) is the only available species in Iran. Public tendency to use herbal remedies and natural products such as synthesized nanoparticles is increasing due to the proof of the destructive side effects of chemical drugs. Nanosilver products have been effective against more than 650 microbe types. This study was aimed at assessing the possibility of green synthesis of silver nanoparticles using *Vaccinium arctostaphylos* aqueous extract and at evaluating its antibacterial properties, as well.

**Materials and Methods:**

In order to synthesize silver nanoparticles, different volumes of *Vaccinium arctostaphylos* aqueous extract (3, 5, 10, 15, and 30 ml) were assessed with different silver nitrate solution concentrations (0.5, 1, 3, 5, and 10 mM) and different reaction time durations (1, 3, 5, 10, and 20 minutes) at room temperature using a rotary shaker with a speed of 150 rpm. Ultraviolet-visible (UV-Vis) spectroscopy, X-ray diffraction analysis (XRD), Fourier transform infrared (FTIR) spectroscopy, and scanning electron microscopy (SEM) were carried out. The antibacterial activity of the aqueous extract and the synthesized nanoparticles was evaluated, as well.

**Results:**

Silver nanoparticle formation process was confirmed with XRD analysis, transmission electron microscopy (TEM), and FTIR spectroscopy. The UV-Vis spectroscopy of silver colloidal nanoparticles showed a surface plasmon resonance peak at 443 nm under optimal conditions (3 ml aqueous extract volume, 1 mM silver nitrate solution concentration, and 3 min reaction time under sunlight exposure). The reduction of silver ions to silver nanoparticles in solution was confirmed, as well. Based on X-ray diffraction analysis, the size of silver nanoparticles was in the range of 7-16 nm. TEM images showed an even distribution of silver nanoparticles, with a spherical shape. FTIR spectroscopy demonstrated the presence of different functional groups of oxygenated compounds such as carboxyl, hydroxyl, and nitrogenous groups. The antibacterial properties of the synthesized nanoparticles were confirmed.

RETRACTED

**Conclusion:**

The synthesized nanoparticles showed more antibacterial properties against gram-positive bacteria (*Bacillus subtilis* and *Staphylococcus aureus*) than gram-negative ones (*Escherichia coli* and *Salmonella enteritidis*).

## 1. Introduction

Strong antibacterial activity is the main objective for the development of nanosilver products as it has been shown to affect more than 650 microbe types [1–3]. Increasing the surface area of silver nanoparticles makes one gram of silver nanoparticles enough to kill bacteria on a surface area of one hundred square meters [4]. There are several ways to reduce Ag^+^ to Ag^0^, including the use of gamma rays, ultraviolet light, heating, electrochemical reduction, and reducing chemicals such as sodium borohydride (NaBH_4_). Although physicochemical methods may have flourishing and well-known net production, however, they are usually expensive, time-consuming, and potentially hazardous to the environment [5].

Unfortunately, many chemical methods of nanoparticle synthesis have disadvantages such as the use of hazardous chemicals and the use of materials with low recyclability and high energy consumption [6]. Rising the environmental concerns over the past decade and the exploration for environmentally friendly synthetic methods have always directed scientists toward biosynthesis which is both economically viable and biologically ecofriendly. Biosynthesis and the use of plants and microorganisms such as bacteria, yeasts, fungi, etc., are among the most widely used methods which have several advantages over chemical and physical methods including environmental compatibility, application of nontoxic and nondestructive environmental materials, the lack of need for temperature, pressure, energy and high-dose chemicals, and also nanoparticle production on a large scale [7–9]. The use of nontoxic chemicals, harmless solvents, and recyclable materials has convinced us to apply biological principles in nanoparticle biosynthesis [10].

Plant chemicals including terpenoids, flavonoids, ketones, aldehydes, amides, and carboxylic acids are directly involved in ion reduction and silver nanoparticle production. Flavones, organic acids, quinones, and water-soluble phytochemicals are responsible for the immediate reduction of silver ions [11].

RETRACTED

Electrostatic attraction between negative charge of bacterial cell and positive charge of nanoparticles [12], Ag ^+^ binding to protein functional groups and their denaturation [13] silver interference with biological macromolecules such as enzymes and DNA through electron emission mechanism [6, 14], and the fact that DNA loses its replication ability [15] determine the antibacterial activity of nanoparticles.

Biosynthesis of silver nanoparticles using sesame seed extract and assessment of the shape of nanoparticles using TEM images showed spherical particles with an average size of 14 nm and silver ion to silver nanoparticle conversion percentage of about 61.99% [16]. The dimension of silver nanoparticles produced using *Cynodan dactylon* extract was estimated to be 30-50 nm in the SEM images and 10-70 nm in XRD spectroscopy [17]. Biosynthesis of silver nanoparticles using Salvia spinosa seed extract and assessment of the shape of nanoparticles using FESEM images showed spherical particles. The nature of particles was crystalline based on XRD spectroscopy. The dimension of silver nanoparticles was estimated to be 19-125 nm based on FESEM imaging, and the diameter of growth inhibition zone against *B. subtilis*, *B. vallismortis*, and *E. coli* was 15 mm, 16 mm, and 12 mm, respectively [18].

Public tendency to use herbal remedies and natural products such as synthesized nanoparticles is increasing due to the proof of the destructive side effects of chemical drugs. More than 60% of Germans and Belgians and 74% of British people prefer natural herbal remedies. Moreover, based on World Health Organization reports, up to 80% of the world's population, especially those of developing countries and poor and remote areas, use medicinal plants. On the other hand, medicinal plants are part of natural resources and a lot of countries have such a resource, though the type, number, and variety of plant species vary based on the conditions and geographical location of each region [19].

The medicinal genus *Vaccinium* from Ericales order and the *Ericaceae* family are popular plants whose medicinal, nutritional, and industrial value is being increased every day. There are 100 species of this genus worldwide of which *Vaccinium arctostaphylos* is the only available species in Iran that has been reported in 6 regions [18].

The most important metabolites in *Vaccinium arctostaphylos* leaves and fruits are phenols, especially cyanosides, which have antioxidant properties. *Vaccinium arctostaphylos* fruits contain 30% sugar, 15.5% protein, and 1.5% fat, with branches containing hexadecanoic acid, tis-pyrene, beta-ionone, and sandracupimaradinin. In Iranian traditional medicine, brewed fruit is recommended for lowering blood sugar and blood pressure [19].

RETRACTED

*Vaccinium arctostaphylos* contains proanthocyanidins which inhibit the adhesion and subsequent proliferation of bacteria, especially *E. coli* and *Helicobacter pylori*, in the epithelium of the urinary tract and gastric mucosa, respectively. Although anthocyanins are found in many other similar fruits, it has shown that the anthocyanidin compounds in *Vaccinium arctostaphylos* have the ability to block bacteria, as well [19].

*Vaccinium arctostaphylos* due to its anticyanocidal compounds helps to form stronger capillaries and reduce platelet adhesion [19]. Vaccinium genus and *Vaccinium arctostaphylos* as its only medicinal species in Iran has economic value.

The antibacterial properties of silver nanoparticles have led to the expansion of its applications in the textile, paint, ceramic, pharmaceutical, agricultural, livestock, food packaging, and cosmetic industries. On the other hand, due to the unique properties of nanoparticles, the use of appropriate production methods in order to achieve nanoparticles with optimal properties, lower cost, and environmental protection is one of the important challenges in the field of nanotechnology. Therefore, based on what was said, the aim of this research was to synthesize silver nanoparticles using *Vaccinium arctostaphylos*, to identify important factors involved in the synthesis of more stable and suitable nanoparticles, and also to investigate the antibacterial effect of the synthesized nanoparticles.

## 2. Materials and Methods

### 2.1. Plant and Extract Preparation

*Vaccinium arctostaphylos* fruit was collected in the summer of 2020 from West Azerbaijan Province, Iran, and subsequently verified by the botany department, Mohaghegh Ardabili University, Iran (Figure 1). Collected fruits were dried in the dark. The extraction was carried out by the maceration method (soaking in water solvent). 100 ml of double-distilled water was added to 10 g of dried sample and subsequently placed on a rotary shaker (Pars Azma, Iran) at a speed of 150 rpm for 24 hours. Following extraction, the extract was filtered using Whatman No. 1 filter paper. Dehydration was performed by anhydrous sodium sulfate. For microbial analysis, the extracts were dissolved in one ml of DMSO, with a dilution rate of 20 mg/*μ*l. To prevent extract decomposition by light and heat, a dark glass container was used to store the extract. Following collection, the resulting extract was stored in the above-mentioned container in the refrigerator [20].

RETRACTED

### 2.2. Nanoparticle Synthesis

In order to synthesize silver nanoparticles, different volumes of *Vaccinium arctostaphylos* aqueous extract (3, 5, 10, 15, and 30 ml) were assessed with different silver nitrate solution concentrations (0.5, 1, 3, 5, and 10 mM) and different time durations (1, 3, 5, 10, and 20 minutes) at room temperature using a rotary shaker with a speed of 150 rpm. Finally, Ag_2_O was obtained from the mentioned treatments according to the following reaction:

(1) $$\begin{array}{c} 2{\text{Ag}}^{+}+2{\text{NO}}_{3}^{-}+2{\text{Na}}^{+}+2{\text{OH}}^{-}\to \text{A}{\text{g}}_{2}\text{O}+2\text{NaN}{\text{O}}_{3}+{\text{H}}_{2}\text{O} \end{array}$$

Ag_2_O precipitate was isolated and washed three times with distilled water. The resulting precipitate was dried at 50°C for 2 hours. Thus, brown Ag_2_O was obtained. Color change to brown and opacity was considered as the first sign of nanoparticle synthesis. Finally, the absorption spectra of all samples were measured at 300 to 800 nm [21]. All experiments were carried out in triplicate.

### 2.3. UV-Vis Spectroscopy

In order to verify the presence of silver nanoparticles, the absorption spectra of the synthesized nanoparticles were taken using the PerkinElmer spectrophotometer (UV/Visible-Lambda 45 model, USA). For this purpose, the treated extract was sampled at different times and the absorption spectra were immediately measured in the wavelength range of 420 to 450 nm, before the sample got dried. This wavelength range corresponds to the silver element, showing fluctuation in the absorption spectrum depending on the size and shape of these particles.

### 2.4. XRD Spectroscopy

XRD spectroscopy was used to investigate the presence of nanoparticles synthesized by fruit extract. Actually, this method investigates the stepwise formation of bioreduced nanoparticles. The crystal structure of the synthesized nanoparticles was examined using an X-ray diffractometer (APD2000 model, Italy), with an X-ray tube with a copper target emitting Cu Ka line with a wavelength of 1.54 Å and Bragg angle of 30° ≤ 2*θ* ≤ 80. Silver nanoparticles formed sharp peaks at 38°, 44°, 67°, and 78° which shows the crystal structure of the characteristic peaks corresponding to (111), (200), (220), and (311) planes, respectively [22]. If the peaks in these four angles are quite sharp and clear, it indicates a favorable interaction between the mineral nanoparticles and the extract, as the nanoparticles get stabilized, giving a characteristic sharp peak. Otherwise, the peaks are weak [23]. On the other hand, the nanoparticle size cannot be obtained directly from the peaks, but its limits can be obtained through the Debye-Scherrer equation [24] as follows:

(2) $$\begin{array}{c} L=K\frac{\lambda }{\beta }\text{CosƟ}, \end{array}$$

where *β* is the width of the peak (full width half maximum), *λ* is the X-ray wavelength at 1.54178 Å (15.4178 nm), *L* is the mean diameter of nanoparticles, *θ* is the angle between radiation and particle plane (diffraction angle here is 40.01), and *K* is a constant which is considered 1 for cubic structures but is 0.9 for silver.

RETRACTED

Nanoparticle size was obtained by averaging the values obtained from three characteristic silver peaks (in the range of 38°, 44°, and 67°). That is, first, the particle size for each sample is calculated at three characteristic silver peaks in the above-mentioned range. Then, the approximate size of the nanoparticles is obtained by getting averages.

### 2.5. FTIR Spectroscopy

For FTIR spectroscopy, 25 ml of 1 mM silver nitrate solution (Merck, Germany) was added to 5 ml of seed extract and kept at 20°C for 24 hours. After completion of the reaction, the sample was centrifuged for 30 minutes at 5000 rpm and then the supernatant was removed. This was repeated three times to ensure. After centrifugation, the sample was dried and the powder was used for FTIR analysis using the PerkinElmer FTIR spectrometer (GX Model, USA). A similar process was conducted for the extract.

### 2.6. Scanning Electron Microscopy (SEM)

In order to specify the size and morphology of the nanoparticles produced using electron microscopy, the reaction mixture was centrifuged three times for 15 minutes at 12,000 rpm. Then, a few drops of the resulting precipitate were dried on a piece of aluminum foil at room temperature, and subsequently, the image was taken by electron microscopy (Philips SEM, CMC-300 KV model, Netherlands).

### 2.7. Assessment of the Antibacterial Activity

Antibacterial effect of silver nanoparticles against gram-positive bacteria including *Staphylococcus aureus* (ATCC25923) and *Bacillus subtilis* (ATCC9372) and gram-negative bacteria including *E. coli* (ATCC25922) and *Salmonella enteritidis* (ATCC13311) was inspected. The bacterial strains were obtained from Zabol Medical Science University.

To evaluate the antibacterial activity by the disk diffusion method [25], a microbial suspension was prepared from a single bacterial colony according to the 0.5 McFarland standards. The bacterial strains were cultured separately on a nutrient agar medium. Eight discs including different concentrations of silver nitrate solution (0.5, 1, 3, 5, and 10 mM), negative control (aqueous extract of the plant), and positive controls (gentamicin and streptomycin antibiotics) were placed on the surface of each plate. 20 *μ*l of each sample was poured onto each disk. The plates were then incubated in an incubator at 37°C. After 24 hours, the inhibition zone was observed. Measurement of the inhibition diameter zone was carried out at least 3 times in each experiment following which the mean was calculated, as well.

RETRACTED

All concentrations of silver nanoparticles were used to specify the minimum inhibitory concentration (MIC). In this test, two positive controls (streptomycin and gentamicin antibiotics) and one negative control (extract) were used.

To determine the minimum bactericidal concentration (MBC), all turbidity-free wells were cultured on Müller-Hinton agar media and subsequently placed in an incubator at 37° for 24 hours. The lowest concentration at which the bacteria did not grow was reported as the minimum bactericidal concentration.

## 3. Results

### 3.1. Biosynthesis of Silver Nanoparticles

The fresh aqueous extract of *Vaccinium arctostaphylos* fruit was pink which changed to dark red after adding 0.001 M silver nitrate solution and exposure to sunlight for 3 minutes (Figure 2).

### 3.2. UV-Vis Spectroscopy

Assessment of the effect of different parameters including silver nitrate solution concentration, aqueous extract volume, reaction time, and the presence of sunlight catalyst on the formation of silver nanoparticles indicated the optimal conditions for nanoparticle synthesis as 1 mM silver nitrate solution, 3 ml of aqueous extract, and 3-minute sunlight exposure. Considering that UV-Vis spectroscopy is an important method for determining the formation and stability of metal nanoparticles in aqueous solution [26], the formation and stability of silver nanoparticles were verified by the UV-Vis spectrum. Therefore, the appearance of a suitable peak at 443 nm indicated the formation of nanoparticles [27]. As silver nanoparticles have adsorption at the range of 400 to 500 nm, the adsorption band of surface plasmon resonance intensification at 443 nm was observed for the synthesized silver nanoparticles (Figure 3(a)).

### 3.3. Assessment of the Effect of Different Extract Volumes on Nanoparticle Synthesis

The effect of different volumes of *Vaccinium arctostaphylos* aqueous extract (3, 5, 10, 15, and 30 ml) on nanoparticle synthesis was investigated in the presence of 1 mM silver nitrate solution, sunlight catalyst, and time exposure of 3 minutes. Based on the results, the optimal volume of 3 ml was selected to follow the experiments (Figure 3(b)).

### 3.4. Assessment of the Effect of Changes in Silver Nitrate Salt Solution Concentration on Nanoparticle Synthesis

The effect of different AgNO_3_ concentrations (0.5, 1, 3, 5, and 10 mM) on silver nanoparticle synthesis was investigated using 3 ml of *Vaccinium arctostaphylos* aqueous extract and time exposure of 3 minutes (Figure 3(c)). It was observed that with increasing AgNO_3_ concentration, the color of the solution gets browner.

RETRACTED

### 3.5. Assessment of the Effect of Reaction Time on Nanoparticle Synthesis

The effect of reaction time (1, 3, 5, 10, 20, and 30 minutes) on silver nanoparticle synthesis was assessed in the presence of 1 mM silver nitrate solution and 3 ml of *Vaccinium arctostaphylos* aqueous extract (Figure 3(d)). It was observed that with increasing the reaction time, there is an opportunity for the reduction phenomenon to be more complete, increasing the number of nanoparticles formed and converting more Ag^+^ into Ag^0^. Moreover, the solution color got darker, and as a result, the maximum wavelength increased with time. Due to the instability of the formed silver nanoparticles, an optimum time is required to complete the reaction, which was obtained as 3 minutes in the present study.

### 3.6. Assessment of the Effect of Sunlight on Nanoparticle Synthesis

Assessment of the effect of sunlight on nanoparticle synthesis in the presence of 1 mM silver nitrate solution and 3 ml of *Vaccinium arctostaphylos* aqueous extract showed that in the absence of light, the reaction is not complete, but when the sample is exposed to sunlight during the autumn and winter days, the reaction gets completed quickly, reducing silver particles (Figure 4).

### 3.7. FTIR Spectroscopy

FTIR spectroscopy was used to identify the active and functional reducing groups of silver ions. The results of the analysis on *Vaccinium arctostaphylos* fruit extract in the presence of silver nitrate solution showed two peaks in 1638 cm^−1^ and 3449 cm^−1^, confirming the presence of oxygenated compounds such as carboxyl, hydroxyl, and nitrogenous groups (Figure 5).

### 3.8. XRD Spectroscopy

XRD spectroscopy of the synthesized silver nanoparticles showed the presence of four sharp peaks at 38°, 44°, 67°, and 78°. The diameter of silver nanoparticles was measured as 11.94 nm in the range of 7-16 nm (Figure 6).

### 3.9. TEM Analysis

TEM analysis of the synthesized silver nanoparticles showed that the particles are nanoscale in size and almost spherical in shape. The size of the synthesized nanoparticles under optimal conditions was measured as 21 nm (Figure 7).

### 3.10. Assessment of the Antibacterial Activity of Silver Nanoparticles

Antibacterial effect of silver nanoparticles against gram-positive bacteria including *Staphylococcus aureus* and *Bacillus subtilis* and gram-negative bacteria including *E. coli* and *Salmonella enteritidis* was inspected. The green synthesized silver nanoparticles using *Vaccinium arctostaphylos* extract had different effects on the diameter of growth inhibitory zone of *E. coli*, *B. subtilis*, and *S. aureus* (*p* < 0.01) (Table 1). While no inhibition zone was observed for *Salmonella* bacterial species, however, the appearance of inhibition zone around the disks for the other three bacterial species verified the antibacterial effect of synthesized silver nanoparticles. An increment of the concentration of synthesized silver nanoparticles increased inhibition zone diameter, as well (Figures 8 and 9). Investigating the minimum inhibitory concentration (MIC) showed more antibacterial activity of silver nanoparticles against *Staphylococcus aureus* as compared to *Escherichia coli* and *Bacillus subtilis* bacterial strains, increasing with rising the concentration and number of nanoparticles (Table 2). Assessment of the minimum bactericidal concentration (MBC) showed more antibacterial activity of silver nanoparticles against *Staphylococcus aureus* as compared to *Escherichia coli* and *Bacillus subtilis* bacterial strains (Table 2).

RETRACTED

## 4. Discussion

The appearance of dark red color in the biosynthesis of silver nanoparticles following reaction with silver ions is an obvious indicator of the reduction of metal ions and the formation of silver nanoparticles which can be due to the changes in the surface plasmon resonance of metal nanostructures [18]. This initial color change which specifies the production of a colloidal suspension of silver nanoparticles [28] can be a good tool to detect the formation of silver nanoparticles in the reaction mixture. Herbal chemical compounds act as the reducing and stabilizing agent to reduce silver ions.

The effect of light on the production of silver nanoparticles varies depending on their size and shape. As the concentration of silver ions increases, the adsorption rate also increases. This is because with increasing the amount of metal ions, more ions are reduced and consequently more nanoparticles will be synthesized [29–31].

Assessment of the effect of different extract volumes on nanoparticle synthesis showed that in smaller plant extract volumes, the intensity of peaks is lower which can be due to decreased amount of reducing agents and thus decreased rate of Ag^+^ ion to Ag^0^reduction. Furthermore, with increasing the concentration of the extract, the intensity of the peaks and the adsorption rate will be increased which can be due to the increase in the number of silver nanoparticles and their agglomeration. Such changes in the adsorption rate may indicate the changes 1in nanoparticle size [32]. In addition, assessment of the optimal concentration among different extract concentrations has shown that increasing the extract concentration will augment nanoparticle synthesis. On the other hand, increasing the concentration of silver nitrate solution has increased nanoparticle synthesis rate, as well [33]. In general, when the volume of the extract increases under constant conditions, more organic material surrounds the nanoparticles. Therefore, the particles settle down, and in very large quantities, the nanoparticles come out of the nanostate which makes the characteristic peak of these nanoparticles no longer visible in the desired range [34].

RETRACTED

Assessment of the intensity of solution discoloration due to the changes in the concentration of silver nitrate solution indicates an increase in the concentration of silver nanoparticles in the solution [35] which is due to the growth of particle size [21]. Spectroscopy analysis results showed that as the concentration of silver nitrate in the solution increases, the particle size and consequently peak intensity increase, as well (Figure 5), while a further increase in silver ion concentration leads to the opposite trend [36]. Increasing silver nitrate solution concentration increases silver nanoparticle synthesis and consequently nanoparticle size and maximum absorption rate [21].

The reaction time is effective in the synthesis and stability of nanoparticles, because if the synthesis process is not complete, the production of nanoparticles will increase over time. Moreover, time is the most significant factor in the verification of the stability of synthesized nanoparticles, because if no increase in the adsorption rate of silver nanoparticles is observed over time, it specifies that the resulting nanoparticles are absolutely stable over time [37].

In FTIR spectroscopy, oxygenated compounds present in the alcoholic and phenolic substances of the extract act as one of the active stabilizing agents to reduce silver nanoparticles [33]. Although the exact mechanism of nanoparticle formation during green synthesis is not yet known, it seems that terpenoids, sugars, phenols, and other plant extract compounds can be used in the synthesis of metal nanoparticles [38].

Adsorption in 1638 cm^−1^ and 3449 cm^−1^ in FTIR analysis corresponds to the affinity of the C-O-H and C = O groups of the extract compounds, the tensile vibrations of the alkyl group, and the C-C bond to a benzene ring. This attribution indicates the presence of the CHO group which can be the main agent to reduce Ag^+^ to Ag^0^ and being converted to CO after reaction.

XRD analysis of silver nanoparticles synthesized in *Euphorbia hirta* extract showed the presence of silver nanoparticles with a diameter of 15-50 nm, but the SEM image confirmed them as 40-50 nm. The results of UV-Vis spectroscopy also showed the absorption peak at 425 nm [39]. It has shown that *Acalypha indica* leaf extract can synthesize silver nanoparticles with a diameter of 20-30 nm and has been effective in inactivating *Escherichia coli* and *Vibrio cholera* bacterial strains [40].

RETRACTED

Green synthesis of silver nanoparticle using aqueous extract of *Fumaria parviflora* and study of its antibacterial and antioxidant properties was achieved. The synthesized silver nanoparticles showed the most absorbance at 430 nm and had a spherical shape with an average size of 10-50 nm. The synthesized nanoparticles had had antioxidant properties with IC_50_ of 21 *μ*g/ml. The results of the antibacterial studies showed that the synthesized silver nanoparticles had had more antibacterial activity against the gram-positive bacteria of *Staphylococcus aureus* than the gram-negative bacteria of *Escherichia coli* [41]. In this research, the synthesized nanoparticles showed more antibacterial properties against gram-positive bacteria than gram-negative, and also, the size of silver nanoparticles was in the range of 7-16 nm that these results were similar to the related research.

Green synthesis and antimicrobial effects of silver nanoparticles were investigated using *Orange blossom* extract, and it was concluded that the formation of silver bioparticles in the range of 400 to 450 nm was demonstrated using a spectrophotometer (UV). The size and morphology of these nanoparticles were determined by a passing electron microscope, and the shape of the spherical particles and their average size was about 5-40 nm [42]. In this research, the size of silver nanoparticles was in the range of 7-16 nm, and also, the shape was the spherical particles that the results are the same.

Although the shape of silver nanoparticles synthesized in the present study is very similar to those of other plants, but their size in this study is smaller than the size of 61 to 117 nm which is reported in a number of studies [43].

At low concentrations of silver nitrate solution, larger nanoparticles are synthesized due to the slower nucleation of nanoparticles. At high concentrations, the final nanoparticles become smaller due to faster nucleation and increasing the number of nuclei in the reaction solution. The size and shape of nanoparticles play a significant role in many of their pharmaceutical applications [44].

The green synthesis of silver nanoparticles was investigated using *Allium paradoxum* plant extract and its antimicrobial activity. It was concluded that the best concentration for the synthesis of silver nanoparticles was 5 mM silver nitrate over a period of 30 minutes [45]. However, in the present study, the best concentration was 1 mM silver nitrate and exposed to sunlight for 3 minutes, which indicates the greater power of *Vaccinium arctostaphylos* plant in the green synthesis of silver particles.

RETRACTED

Silver has long been known for its antibacterial properties. In fact, silver nanoparticles exhibit such properties against aerobic and anaerobic bacteria due to the release of silver ions. Binding of these particles to sulfur-containing proteins on the surface of bacterial membranes allows the entry and subsequent changes in the morphology and respiratory chain of bacteria which finally leads to the death of the foreign agent by affecting the cell death process [46].

The effect of nanoparticles on the cells of living organisms depends on their diameter, size, and shape [47]. Larger nanoparticles are more toxic due to their easier absorption and larger surface area. Furthermore, the release rate of silver ion is increased as the size of silver nanoparticles decreases. Therefore, the toxicity of silver nanoparticles depends on their size and the amount of silver ion release rate [48]. However, other factors such as crystallinity, stabilizing reagents, and environmental factors including pH, the presence of ligands, and divalent cations in solution and macromolecules have also been considered significant [49]. In general, silver nanoparticles, due to their smaller size, have a greater contact surface with the environment and microorganisms. This increases their biological and chemical activities and consequently their impact on cell membranes [50–52]. At low concentrations, due to the small number of nanoparticles, the degree of interaction of the nanoparticles with the bacterial cell membrane is less and thus the inhibitory effect of nanoparticles is low and the diameter of the inhibition zone is small. For this reason, a balanced concentration of nanoparticles is always desirable to inhibit the bacterial growth [25].

The antimicrobial effect and effective parameters on the stability of silver nanoparticles synthesized using *Mentha pulegium* were investigated, and it was concluded that the distribution of nanoparticles with spherical shapes was almost uniform. The study of the effect of different variables in the synthesis of these nanoparticles has shown that the volume of the extract is 3 ml, the concentration of silver nitrate salt is 1 mM, and the reaction time of 10 minutes in sunlight is the best conditions to achieve maximum stability of silver nanoparticles [53]. In the present research, the UV-Vis spectroscopy of silver colloidal nanoparticles showed a surface plasmon resonance peak at 443 nm under optimal conditions (3 ml aqueous extract volume, 1 mM silver nitrate solution concentration, and 3 min reaction time under sunlight exposure) that the optimal conditions are the same with related research.

RETRACTED

The major property of silver nanoparticles is their antibacterial activity which is used in wound dressing, skin wound ointments, disinfectants, and medical instrument coatings. These nanoparticles shorten the duration of the wound healing process by reducing the activity of metalloproteases and boosting the apoptosis of neutrophils, making the appearance of scars more natural. In addition, they will be effective in better collagen orientation and enhance the mechanical strength of the tissues. Assessment of wound dressings has shown that silver usage for similar applications does not cause toxicity or adverse effects on human cells. Recent studies have also demonstrated that the use of silver nanoparticles in skin ointments causes silver penetration into the wound bed, absorption by the epidermal cells of the wound margin, accumulation in the wound debris, and eventually transfer to the peripheral circulatory system which helps the wound healing process and prevent infection [54].

In this study, the antimicrobial activity of *Vaccinium arctostaphylos* aqueous extract and its synthesized silver nanoparticles were evaluated on four bacterial strains. The results showed that the nanoparticles in concentrations used had stronger antimicrobial effects than the extract itself which was concentration dependent in both the extract and the nanoparticle solution. While silver nanoparticles had more antimicrobial activity against gram-positive bacteria, gram-negative bacteria showed resistance to silver nanoparticles.

To date, different reports have been presented about the greater effect of silver nanoparticles on gram-negative bacteria [3, 55–57] or gram-positive bacteria [29, 58–60] and even the lack of difference between gram-positive and gram-negative ones [61].

Some reports have attributed the difference in the response of gram-positive and gram-negative bacteria to silver nanoparticles to the difference in their cell wall structure [48, 62], and some reports have pointed to the effect of silver nanoparticles on the structure of the bacterial cell membrane and the reduction of cell leakage and ultimately the bacterial death [58]. However, the effect of silver nanoparticles on cell membrane structure and reduction of cell leakage (extracellular vesicle production) seems to be greater. However, if the antibacterial effect of silver nanoparticles is related to the peptidoglycan layer (a specific feature of the membranes of bacterial species which is not observed in mammalian cells), the use of silver nanoparticles as an antibacterial agent will be easier and more specified.

RETRACTED

All domains of life on Earth, including gram-negative and gram-positive bacteria as well as eukaryotic organisms, actively secrete nanometer-sized vesicles (conserved intercellular evolutionary components). These structures are round, bilayer containing biologically active substances such as proteins, lipids, nucleic acids, and metabolites that can act as secretory systems for the secretion of toxins, enzymes, and pathogens in bacteria. On the other hand, these structures can increase the survival rate in bacteria. Resistance to antibacterial compounds can take place by releasing these vesicles at all stages of the bacterial growth. Actually, the production of these vesicles can augment the survival of bacteria when attacked by phages. These structures can remove antibacterial agents such as supplements and antibiotics, as well [63]. It has even been reported that *S. aureus* extracellular vesicles contain beta-lactamase which causes the survival of ampicillin-sensitive gram-positive and gram-negative bacteria in the presence of ampicillin [64–66] [60–62]. Evidence also suggests that the secretion of extracellular vesicles is a completely conserved evolutionary process in gram-positive bacteria [64, 67] [60, 63]. Therefore, the higher sensitivity of gram-positive bacteria as compared to gram-negatives in this study may be due to the role of silver nanoparticles in further reducing the production of extracellular vesicles in gram-positive bacteria.

In general, the mechanism of antimicrobial activity by silver nanoparticles is related to their ability to cross cell membranes and how they affect cellular components such as DNA, proteins, and others which ultimately disrupt DNA replication and the activity of proteins and bacterial enzymes, leading to bacterial death [33].

The most common mechanism for the antibacterial effect of silver nanoparticles is the ionic release of silver and the inactivation of thiol groups in enzymes, which inactivate bacterial enzymes. The released silver ions inhibit bacterial DNA replication, damage cell cytoplasm, reduce adenosine triphosphate (ATP) levels, and eventually kill bacterial cells. Increasing the surface to volume ratio of nanoparticles increases the binding level of nanoparticles to the bacterial cell. This action increases the release of silver ions to the bacteria and thus improves the antibacterial effect of silver [68].

Nanotechnology is an attractive field of research for human beings due to the production of nanoparticles in different sizes, shapes, chemical compositions and distributions, and its many applications. The fabrication, manipulation, and use of metal nanoparticles are of great importance due to their reduced dimensions and consequently their unique thermal, optical, and electronic properties [69].

RETRACTED

Today, the synthesis of silver nanoparticles is very common due to their many applications in various fields. The synthesis of these nanoparticles is done through physical, chemical, and biological methods. The biological method is preferable to the other two methods due to its compatibility with the environment and its low cost. Green nanoparticle production is a nature-friendly method that uses natural solvents [70].

Past studies in the field of nanoparticles show that due to the lack of a logical model of the interaction of these particles with biological molecules, so far from trial and error methods, the properties of a nanoparticle and its effects on the reaction medium and molecules are present. They found out in that environment. Due to the entry of these particles into plants and animals, and especially their increasing use in products used by humans, it seems necessary to study the effects of these particles on molecules and biological hosts [71].

## 5. Conclusion

The biosynthesis of silver nanoparticles by *Vaccinium arctostaphylos* aqueous extract was determined and confirmed by UV-Vis spectroscopy and transmission electron microscopy. The silver nanoparticles obtained at the reaction time of 3 minutes had an average size of 12 nanometers and an almost spherical shape. Synthesized silver nanoparticles showed more antibacterial activity against gram-positive bacteria than gram-negative bacteria, especially against *Staphylococcus aureus*.

In general, our results showed that *Vaccinium arctostaphylos* aqueous extract has a good potential to produce silver nanoparticles. Both the extract and the synthesized nanoparticles have significant biological potential. In case additional studies are carried out and side effects are assessed and the conditions are optimized, they can be used in food, pharmaceutical, and agricultural industries and in the near future as natural antioxidant supplements with more efficacy.

## Figures and Tables

**Figure 1:** Morphological characteristics of leaves and fruit of *Vaccinium arctostaphylos* L.

**Figure 2:** Color change of fruit extract (a) before and (b) after adding silver nitrate solution.

**Figure 3:** (a) UV-Vis spectrum under optimal conditions; (b) UV-Vis spectra of silver nanoparticles using different volumes of *Vaccinium arctostaphylos* aqueous extract (3, 5, 10, 15, and 30 ml), in the presence of 1 mM silver nitrate solution, sunlight catalyst, and time exposure of 3 minutes; (c) the effect of different AgNO_3_ concentrations on silver nanoparticle synthesis using 3 ml of *Vaccinium arctostaphylos* aqueous extract; (d) the effect of reaction time on nanoparticle synthesis using *Vaccinium arctostaphylos* aqueous extract.

RETRACTED

**Figure 4:** The effect of the presence and absence of 3-minute sunlight exposure on nanoparticle synthesis using *Vaccinium arctostaphylos* aqueous extract.

**Figure 5:** FTIR spectrum of silver nanoparticles synthesized under optimal conditions.

**Figure 6:** XRD spectrum of silver nanoparticles synthesized under optimal conditions.

**Figure 7:** TEM analysis of silver nanoparticles synthesized under optimal conditions.

**Figure 8:** Inhibition zone diameter of different concentrations of silver nitrate solution synthesized in *Vaccinium arctostaphylos* aqueous extract. Similar letters indicate no significant difference.

**Figure 9:** Disc diffusion test using 5 different concentrations of silver nitrate solution ((a) 10 mM; (b) 5 mM; (c) 3 mM; (d) 1 mM; (e) 0.5 mM). The aqueous extract of the plant was considered as the negative control, and gentamicin and streptomycin antibiotics were considered as the positive control.

**Table 1:** Diameter variance analysis of inhibitory zone of green synthesis of silver nanoparticles using *Vaccinium arctostaphylos* extract against different bacterial agents.

S.O.V	df	MS		
		*E. coli*	*B. subtilis*	*S. aureus*
Source	6	113.857^∗∗^	147.969^∗∗^	141.714^∗∗^
Error	14	0.857	1	0.857
Total	20			

^∗∗^Significant at the level of one percent.

**Table 2:** MBC and MIC test analysis against *Staphylococcus aureus*, *Escherichia coli*, and *Bacillus subtilis* bacterial strains.

Cases under review	*E. coli*		*B. subtilis*		*S. aureus*	
	MIC (*μ*g/ml)	MBC (*μ*g/ml)	MIC (*μ*g/ml)	MBC (*μ*g/ml)	MIC (*μ*g/ml)	MBC (*μ*g/ml)
Extract	—	—	—	—	—	—
AgNO_3_	100 ppm	200 ppm	100 ppm	200 ppm	12.5 ppm	25 ppm

## Data Availability

No data were used to support this study.
